# Multiple Traffic Target Tracking with Spatial-Temporal Affinity Network

**DOI:** 10.1155/2022/9693767

**Published:** 2022-05-23

**Authors:** Yamin Sun, Yue Zhao, Sirui Wang

**Affiliations:** ^1^School of Architecture & Civil Engineering, Xi'an University of Science & Technology, Xi'an 710054, China; ^2^Postdoctoral Research Station on Civil Engineering, Xi'an University of Science & Technology, Xi'an 710054, China; ^3^School of Civil Engineering & Architecture, Xi'an University of Technology, Xi'an 710048, China; ^4^Shaanxi Transportation Holding Group Co., Ltd., Xi'an 710000, China

## Abstract

Traffic target tracking is a core task in intelligent transportation system because it is useful for scene understanding and vehicle autonomous driving. Most state-of-the-art (SOTA) multiple object tracking (MOT) methods adopt a two-step procedure: object detection followed by data association. The object detection has made great progress with the development of deep learning. However, the data association still heavily depends on hand crafted constraints, such as appearance, shape, and motion, which need to be elaborately trained for a special object. In this study, a spatial-temporal encoder-decoder affinity network is proposed for multiple traffic targets tracking, aiming to utilize the power of deep learning to learn a robust spatial-temporal affinity feature of the detections and tracklets for data association. The proposed spatial-temporal affinity network contains a two-stage transformer encoder module to encode the features of the detections and the tracked targets at the image level and the tracklet level, aiming to capture the spatial correlation and temporal history information. Then, a spatial transformer decoder module is designed to compute the association affinity, where the results from the two-stage transformer encoder module are fed back to fully capture and encode the spatial and temporal information from the detections and the tracklets of the tracked targets. Thus, efficient affinity computation can be applied to perform data association in online tracking. To validate the effectiveness of the proposed method, three popular multiple traffic target tracking datasets, KITTI, UA-DETRAC, and VisDrone, are used for evaluation. On the KITTI dataset, the proposed method is compared with 15 SOTA methods and achieves 86.9% multiple object tracking accuracy (MOTA) and 85.71% multiple object tracking precision (MOTP). On the UA-DETRAC dataset, 12 SOTA methods are used to compare with the proposed method, and the proposed method achieves 20.82% MOTA and 35.65% MOTP, respectively. On the VisDrone dataset, the proposed method is compared with 10 SOTA trackers and achieves 40.5% MOTA and 74.1% MOTP, respectively. All those experimental results show that the proposed method is competitive to the state-of-the-art methods by obtaining superior tracking performance.

## 1. Introduction

Traffic target tracking in dynamic traffic scenes is a fundamental problem in intelligent transportation, particularly for vehicle autonomous driving to perceive the directions of other vehicles and pedestrians [1]. It is not only useful for information sharing between vehicles and users, but also helpful for realizing data interaction in intelligent transportation system. The goal of traffic target tracking is to follow the trajectories of vehicles or pedestrians as they move in video sequences. In recent years, vision-based multiple vehicle tracking is widely used in autonomous driving, electronic police, checkpoint monitoring, and road monitoring [2, 3].

With the development of deep-learning, the multiple objects tracking (MOT) also benefits from the representational power of deep neural network. It is a competitive choice for appearance modelling in MOT to extract complex and abstract features. Since pedestrians in videos have discriminative appearances with different colors and types of cloth, and the motion follows the social force model that typically uses the first or second order motion to predict the object states, the deep learning-based multiple pedestrian tracking algorithms achieve good performances. Different from the pedestrians in videos, the vehicles often have similar appearance with limited shape and color variation. In addition, the motion often changes drastically with sudden acceleration or brakes. Hence, the deep leaning-based multiple vehicles tracking algorithms tend to perform worse than multiple pedestrian tracking algorithms. This motivates researchers to not only simply rely on the deep neural network to learn rich representation of input, but also pay more attention on how to fully exploit deep learning in both association affinity computation and data association process.

The state-of-the-art MOT approaches conform to the tracking-by-detection framework, which includes two core steps: (1) object detection in video sequences and (2) data association between detections over video sequences to form long trajectories. Traditional MOT methods which follow the tracking-by-detection framework often use publicly available detections and mainly focus on how to construct a robust data association module to gain tracking performance. For data association, association affinity computation between detections is calculated by multiple cues, such as appearance, location, and topology [4]. These methods mainly pay attention to spatial or appearance features in two adjacent frames, ignoring the features of temporal variations from the history trajectory in consecutive frames.

Recently, with the help of the transformer's powerful self-attention mechanism for features encoding [5], the 2D tracking can achieve amazing performance. The self-attention and position mechanism in transformer model can effectively encode the correlation of tracked objects. The corresponding position information is also recorded, which is useful to handle the issues such as occlusion and disappearance of the tracked objects. Hence, the content-adaptive property and position encoder ability of transformer motive us to introduce it into MOT, aiming to fully capture and encode the spatial and temporal information from the detections and the tracklets of tracked targets in MOT task. However, transformer model lacks the properties of translation invariance and local correlation, which are two key inherent properties of convolution neural network (CNN). The limited receptive field of CNN makes it difficult to capture global information, while the transformer can model long-range dependencies. Therefore, it is a good choice to combine CNN and transformer together, so that the network can inherit the advantages of CNN and transformer and capture global and local features at large.

Motived by the ideal performance of transformer's powerful self-attention mechanism for feature encoding, a spatial-temporal encoder-decoder affinity network for multiple traffic target tracking is proposed in this study. As shown in Figure 1, a CNN feature extractor (Resnet-50) is first used to learn abstract and low resolution features from the detections images. Then, a spatial-temporal encoder-decoder affinity network is designed to process and aggregate the spatial and temporal information of the tracked objects in different frames. The spatial-temporal encoder-decoder affinity network mainly consists of two parts: the transformer-based spatial-temporal two-stage encoder subnetwork and the spatial transformer decoder subnetwork for association affinity computation. In the two-stage encoder subnetwork, the feature maps of candidate detections and the tracked targets captured by CNN feature extractor are encoded separately to capture the spatial correlation and temporal discriminative history features at the image level and tracklet level. In the spatial transformer decoder association network, the results from the two-stage transformer encoder subnetwork are fed back as keys to guide the association computation for the attention weights of the object query and the tracklet query. This is useful for fully capturing and encoding the spatial and temporal information from the detections and the tracklets of tracked targets. After achieving the assignment association matrix between the candidate detections and the existing tracklets, the final tracking results are achieved by performing the Hungarian algorithm to solve the association problem between the detections and the tracked objects.

In summary, the main contributions of the proposed method are as follows:

1. A cascade association network, consisting of a transformer-based spatial-temporal two-stage encoder subnetwork and a spatial transformer decoder data association subnetwork, is designed for online multi-traffic target tracking.
2. The two-stage transformer encoder framework is designed to encode candidate detections and the tracked targets to capture the spatial correlation and temporal history trajectories features at the image level and tracklet level, respectively.
3. A spatial transformer decoder association network is designed for data association in online tracking, where the results from the two-stage transformer encoder subnetwork are fed back as keys to guide the association computation for the attention weights of the object query and the tracklet query, aiming to fully capture and encode the spatial and temporal information from the detections and the tracklets of tracked targets.

## 2. Related Works

With the representational power of deep neural network, the deep-learning-based MOT method has shown significant improvement in extracting complex and abstract features. In this section, we mainly present some relevant literature regarding deep-learning-based MOT algorithms.

The state-of-the-art MOT methods that follow the tracking-by-detection framework often divide the MOT into two procedures: object detection by detectors in each frame and data association to link the detections in consecutive frames to generate the trajectories. In tracking-by-detection MOT, with the detections provided by a predefined detector, data association plays a key role in improving the tracking performance. The function of association affinity is to correctly associate tracked target with detections and it is always calculated by multiple cues such as appearance, location, and topology. With the powerful representational ability of deep neural network, many researchers exploit deep neural network for appearance modelling. Liu et al. [6] used a Siamese network to construct multi-level similarity model for thermal infrared object tracking. Scheidegger et al. [7] adopted a deep neural network to train detection and to estimate the distance between the objects for multi-object tracking. It is useful for eliminating ambiguous features in appearance modelling. Yuan et al. [8] proposed a self-supervised learning-based tracker by devising deep correlation framework for feature extraction, which is helpful for gaining the feature representational ability and reducing the overfitting risk. In [9], a metric learning model is introduced into correlation filters framework, which is useful for solving the fixed scale and noise interference for visual tracking. Though the above deep-learning-based tracking methods can achieve good performances, directly using deep neural network for appearance modelling in multiple vehicle tracking may limit the tracking performance since vehicles are often have similar appearances. In our study, the deep neural network is not only used for context feature extraction, but also used to guide data association between the detections and the tracked objects.

Several data association methods were presented to improve the MOT performance in recent studies. Bea and Yoon [10] introduced transfer learning into a revised Siamese network to learn discriminative deep appearance features for robust tracking. Schulter et al. [11] designed a network-flow-graph-based data association model via backpropagation for multiple object tracking. Li et al. [12] regarded the MOT as a graph optimization problem and designed appearance and motion graph networks as solution. He et al. [13] proposed a general undirected graph model to solve the association problem via graph matching between tracklet and detection graphs. Muresan et al. [14] devised a robust data association method for pedestrian tracking in thermal images, where five Siamese networks were used to construct a data-driven and appearance-based association score for tracking. The existing data association methods in MOT mainly rely on a graph-based optimization or network flow to achieve the association cost between the detections and the tracklets. These methods always focus on the local relationship by static graphs and ignore the history tracklets information, making it difficult for tracker survival in severe occlusion. In our study, these problems are addressed by designing a two-stage transformer encoder model to encode history trajectories and the detection information in tracklet level and image level.

Recently, inspired by its remarkable success in natural language processing (NLP), transformer modules are transplanted from the NLP to computer vision. This module is a self-attention-based architecture with the ability to handle long sequence data, in which the attention mechanism is a key idea and plays an important role in the transformer model [5]. The transformer module has wide applications in image classification, object detection, pose estimation, person re-identification, action recognition, object tracking, and other computer vision areas. Following the success of transformer modules introduced in detection and tracking tasks, Xu et al. [15] proposed a transformer-based architecture for multi-object tracking, in which dense queries were introduced in a double-decoder network to robustly infer the heatmap for the tracked targets. Meinhardt et al. [16] proposed an encoder-decoder transformer framework for MOT, which achieved state-of-the-art performance. In [17], a powerful transformer network is adopted for 3D single object tracking, which uses the transformer module to compute attention weights for features. All these methods gain tracking performance via transformer attention mechanism. In the present study, we propose a spatial-temporal encoder-decoder affinity network for multiple traffic target tracking, in which a transformer-based spatial-temporal two-stage encoder model is designed to extract context information from the detections and the tracklets. Thus, the proposed method introduces the long history trajectory information into the feature encoder and decoder procedures with self-attention and position mechanism in transformer model, which is useful in handling the occlusion in online tracking.

## 3. Proposed Network

### 3.1. Problem Formulation

Figure 1 shows the proposed MOT tracking, which follows the tracking-by-detection framework. A detection set *𝔻*_*t*_={*D*_*t*_^1^, ⋯, *D*_*t*_^*N*^} is provided by a predefined detector in online tracking at each frame *t*. The linked detections from frames 1 to *t* − 1 formulate a tracklet set *𝕋*_*t*−1_={*T*_*t*−1_^*j*^}_*j*=1_^*M*_*t*−1_^. Then, the online MOT performs data association between the detection set *𝔻*_*t*_ and the tracklet set *𝕋*_*t*−1_ in frame *t* to achieve the final trajectories *𝕋*_*t*_={*T*_*t*_^*j*^}_*j*=1_^*M*_*t*_^. The last detection on one trajectory is the tracked object. In the algorithm, the online MOT aims to match the current detections and the tracked objects in each frame *t*. With *N*_*t*_ detection *𝔻*_*t*_={*D*_*t*_^1^, ⋯, *D*_*t*_^*N*_*t*_^} and *M*_*t*−1_ tracklets *𝕋*_*t*−1_={*T*_*t*−1_^*j*^}_*j*=1_^*M*_*t*−1_^, the algorithm first uses the convolutional neural network (CNN) to extract the visual feature of the *N*_*t*_ candidate detections. Then, the spatial transformer encoder module is used to encode the detections at the image level. The temporal transformer encoder module is used to extract the discriminative information from the tracklets of the tracked objects at the tracklet level. Finally, the spatial transformer decoder module is devised to compute assignment association matrix for correctly associating the candidate detections and the existing tracklets. The final tracking results are achieved by performing the Hungarian algorithm to solve the association problem between the detections and the tracked objects.

For each tracklet *T*_*t*−1_^*j*^ ∈ *𝕋*_*t*−1_ in frame *t*, the best candidate detection is determined by finding the *D*_*t*_^*i*^ to maximize the association affinity *A*(*T*_*t*−1_^*j*^, *D*_*t*_^*i*^), where *A*(*·*) denotes the affinity score between the tracklet and the candidate detection. By considering all tracklets and the detections in frame *t*, the association can be regarded as an optimization problem and is expressed as follows:

(1) $$\begin{array}{c} \max\sum_{i=1}^{N_{t}}\sum_{j=1}^{M_{t-1}}\beta_{t}^{ij}A\left(T_{t-1}^{j},D_{t}^{i}\right), \end{array}$$

where *β*_*t*_^*ij*^ ∈ {0,1}, ∀*i*=1, ⋯, *N*_*t*_; *j*=1, ⋯, *M*_*t*−1_ denotes the association between detection *𝔻*_*t*_={*D*_*t*_^1^, ⋯, *D*_*t*_^*N*_*t*_^} and tracklets *𝕋*_*t*−1_={*T*_*t*−1_^*j*^}_*j*=1_^*M*_*t*−1_^ in frame *t*. If the detection *D*_*t*_^*i*^ is associated with tracklet *T*_*t*−1_^*j*^, *β*_*t*_^*ij*^=1; otherwise, *β*_*t*_^*ij*^=0.

### 3.2. Two-Stage Transformer Encoder Model

Benefiting from the good performance of a CNN-based transformer framework [18], we first utilize a CNN named Resnet-50 backbone as a feature extractor. Figure 1 shows the CNN backbone; the first three blocks are adopted to extract feature maps for candidate detections at each frame. Then, the two-stage transformer encoder framework is used to encode the feature maps of the detections and the tracklets. In the first stage, the spatial-transformer encoder module is used to encode the spatial image information, which deals with the patch tokens at the image level. In the second stage, the temporal transformer encoder module is used to encode the history trajectory information, which processes the image tokens at the tracklet level. The transformer follows a query-key encoder-decoder framework, in which the encoder generates keys and the decoder inputs task-specific queries [19]. The transformer consists of multi-head self-attention (MHA) layers and feed-forward network. If the input key and query are the same, the MHA is called self-attention; otherwise, it is called cross-attention. After performing the two-stage transformer encoder module, the keys for decoder can be achieved. Then, the features maps extracted by CNN for detections are regarded as the object query, and the detection features from the existing tracklets are concatenated to form the tracklet query. Both object query and tracklet query serve as the input for the decoder module. The assignment association matrix used to associate the candidate detections and the existing tracklets is generated by performing the spatial transformer decoder module. Finally, the Hungarian algorithm [20] is used to solve the association problem between the detections and the tracked objects.

#### 3.2.1. Image-Level Feature Extraction with the Spatial Transformer Encoder Module

After the CNN backbone (Resnet-50) is used to extract features maps for each detection at frame *t*, the corresponding feature maps *ε*_*t*_=*f*{*D*_*t*_^*i*^}^*i*=1,⋯,*N*_*t*_^ for the detection set are formed. Then, the spatial transformer encoder module (STE) is utilized to extract detections features at image level. For each feature map *f*{*D*_*t*_^*i*^} of detection *D*_*t*_^*i*^ with size *H* × *W* generated from Resnet-50, it is first divided into small patches *x*_*t*_^*i*^. Then, these spatial patches are fed into the spatial-transformer module to learn discriminative representation in spatial dimension at the image level.

With the small patches in each frame, the general vision transformer [5] is followed to perform the feature encoder among all spatial patches. First, the spatial patches *x*_*t*_^*i*^ are flattened into one-dimension tokens and are then embedded through a linear embedding layer as follows:

(2) $$\begin{array}{c} z_{0}=\left[x_{t}^{1}E;x_{t}^{2}E;\cdots x_{t}^{i}E;\cdots x_{t}^{N}E\right]+E_{\text{pos}}, \end{array}$$

where the output *z*_0_ refers to spatial embedded feature with positional embedding, *x*_*t*_^*i*^ ∈ *ℝ*^*N*×(*p*^2^*·C*)^ is the spatial patches, (*p*, *p*) is the size of each spatial patch, *N*=*H* × *W*/*p*^2^ is number of the patches, and *C* denotes the dimension of spatial embedding. *E* ∈ *ℝ*^*p*^2^×*C*^ is a linear projection matrix, and *E*_*pos*_ ∈ *ℝ*^(*N*+1)×*C*^ is the position embedding.

Subsequently, the spatial embedded feature *z*_0_ is fed to the transformer encoder module as follows:

(3) $$\begin{array}{c} z_{l}^{\prime }=MHA\left(LN\left(z_{l-1}\right)\right)+z_{l-1},\;l=1,2,\cdots ,L, \end{array}$$

(4) $$\begin{array}{c} z_{l}=MLP\left(LN\left(z_{l}^{\prime }\right)\right)+z_{l}^{\prime },\;l=1,2,\cdots ,L, \end{array}$$

(5) $$\begin{array}{c} Y_{\text{key}}^{de}=LN\left(z_{L}\right). \end{array}$$

The transformer encoder module comprises multi-head self-attention function (MHA) in equation (3) and the multi-layer perceptron blocks (MLP) in (4) with *L* layers, as shown in Figure 2. Layer normalization operator LN is applied before every block. For layer of *l* = 1, the (3) is initialized by the spatial embedded feature *z*_0_, which is computed in (2). By performing the MHA for *z*_0_ in (3), the output of MHA *z*_1_′ is fed to MLP in (4). Then, the output of the MLP *z*_1_ acts as the input of MHA in (3) for next time iteration. After iteration L times of MHA and MLP in (3) and (4), the final output is the concatenation of *h* attention head results. *Y*_key_^*de*^ in (5) with normalization operator (LN) is the key for the decoder module to guide computation the association affinity matrix for correctly associating the candidate detections and the existing tracklets.

#### 3.2.2. Tracklet-Level Feature Extraction with Temporal Transformer Encoder Module

Since the tracklets of the same object are closer than those of different identities in consecutive frames, the history tracklets of the tracked target may provide efficient temporal features to solve the occlusion or object disappear issues. Hence, to fully exploit the temporal information of the tracked objects in different frames for association affinity computation, a temporal transformer encoder (TTE) module is devised to encode the features of the tracked target in tracklet level. After performing the STE module to encode the detections at each individual frame in image level, the output of the spatial transformer *z*_*L*_ is encoded and flattened as a vector *z*. For the *t* − *th* frame, the existing tracklet set *𝕋*_*t*−1_={*T*_*t*−1_^*j*^}_*j*=1_^*M*_*t*−1_^ is formulated by linking detections from frames 1 to *t* − 1. By concatenating the spatial feature vectors {*ε*_*t*−*T*_, *ε*_*t*−*T*+1_, ⋯, *ε*_*t*−1_} of the tracked target tracklets from the past *t* − 1 frames, the input Ξ_*t*−1_={*ε*_*t*−*T*_, *ε*_*t*−*T*+1_, ⋯, *ε*_*t*−1_}, Ξ ∈ *ℝ*^(*t* − 1)×*p*^2^*·C*^ for the temporal transformer module is achieved, where *ε*_*t*−1_={*z*_*k*_^*i*^}_*k*=1,⋯,*t*−1_^*i*=1,⋯,*N*_*k*_^, *k* is the frame index, and *N*_*k*_ is the number of the detections in frame *k*. The temporal positional embedding *E*_*Tpos*_ ∈ *ℝ*^(*t* − 1)×*C*^ is first performed to maintain the frame position information. Then, the temporal embedded feature Ξ_*t*−1_ is fed to the TTE module, which has the same architecture with STE module and consists of MHA and MLP blocks. The output of the TTE module *Y*_key_^*tr*^ is the key for the decoder module to construct the association affinity matrix for correctly associating the candidate detections and the existing tracklets.

### 3.3. Spatial Transformer Decoder Module for Computing Association Affinity Matrix

The proposed spatial transformer decoder (STD) module used for constructing association affinity matrix is shown in Figure 3. First, the feature maps *ε*_*t*_ and Ξ_*t*−1_ extracted for detections and tracklets by the Resnet-50 network are used as the object queries and tracklet queries. Then, the keys for STD are achieved by feeding back the results of *Y*_key_^*de*^ and *Y*_key_^*tr*^ from the two-stage transformer encoder module, which is described in Section 3.2. With the queries and keys, the STD module is used to generate the assignment matrix *A*_*t*_ to correctly associate the detections and the tracklets at each frame *t*. The STD module first uses the MHA to encode the object queries and tracklet queries, respectively. Then, the attention weighted object queries and tracklet queries are represented as *F*_*att*_^*de*^ ∈ *ℝ*^*N*_*t*_×1×*C*^ and *F*_*att*_^*tr*^ ∈ *ℝ*^(*t* − 1)×*M*_*t*−1_×*C*^. This process is similar to that of the encoder in Section 3.2. For the data association of the *N*_*t*_ detections and the *M*_*t*−1_ tracked objects in frame *t*, if the number of detections *N*_*t*_ is larger than *M*_*t*−1_, the virtual source is introduced to address the case that initiates the detections to new tracklets in frame *t*, and the number of virtual sources is *M*_*v*_=*N*_*t*_ − *M*_*t*−1_. After adding the virtual source, a new tracklet embedding *F*_*att*_^*tr*′^ ∈ *ℝ*^(*t* − 1)×(*M*_*t*−1_+*M*_*v*_)×*C*^ is formed. Then, multihead cross attention is performed for *F*_*att*_^*tr*′^ and *F*_*att*_^*de*^. Next, multi-layer perceptron and normalization layer follows to generate the output tensor *ℝ*^*N*_*t*_×(*M*_*t*−1_+*M*_*v*_)×*C*^, which denotes the matching between the tracklets and the detections. Finally, the output of the spatial transformer decoder goes through linear and softmax layers to generate the assignment matrix *A*_*t*_ ∈ *ℝ*^*N*_*t*_×(*M*_*t*−1_+*M*_*v*_)^.

### 3.4. Data Association

After achieving the assignment matrix *A*_*t*_ ∈ *ℝ*^*N*_*t*_×(*M*_*t*−1_+*M*_*v*_)^ for the detections and existing tracklets at each frame *t*, the Hungarian algorithm [20] is used to solve the association problem between the detections and the tracked objects. This is done by maximizing the affinities between the current frame detections and the detections already assigned to the tracked targets in previous frames. With the data association, the final tracking results are achieved by solving the maximizing problem in (1). The unmatched detections in each frame are stored as a nonmatched detection set, which is used to initiate new targets or to recover occlusion. Similarly, the unmatched tracklets are remained as a nonassociated tracklet set, which is regarded as the cases that the tracked objects exit the scene or are occluded. The corresponding visual features and bounding boxes of the unmatched detections and unassociated tracklets are all stored for next frame data association. Finally, a new tracklet is born when the detection in nonmatched detection set is associated with other detections in five consecutive frames. Otherwise, the detection is removed when it is not association with any detection or the tracklet exceed five frames. A tracklet is killed in nonassociated tracklet set if the number of frames for its tracklet is not associated with any detection exceeding five consecutive frames.

### 3.5. Loss Function

When training the proposed network, the cross-entropy loss is taken as the loss function to optimize the network. For the *N*_*t*_ detection and *M*_*t*−1_ tracklets at each frame *t* in each training iteration, the cross-entropy loss *ℓ* is defined as follows:

(6) $$\begin{array}{c} \ell =-\frac{1}{N_{t}}\sum_{i=1}^{N_{t}}y_{i}\log\left(a_{i}\right)+\frac{\lambda }{M_{t-1}}\sum_{j=1}^{M_{t-1}}y_{j}\log\left(\frac{1}{1+e^{-{a_{j}}^{\prime }}}\right)+\frac{\lambda }{M_{t-1}}\sum_{j=1}^{M_{t-1}}\left(1-y_{j}\right)\log\left(\frac{e^{-{a_{j}}^{\prime }}}{1+e^{-{a_{j}}^{\prime }}}\right), \end{array}$$

where *y*_*i*_ and *y*_*j*_ are IDs of the detections and the tracklets in frame *t*, *a*_*i*_ is the row element of *A*_*t*_, and *a*_*N*_*t*__={*a*_*j*_′}, *λ* is a weighting coefficient.

## 4. Experiments and Results

### 4.1. Datasets

To validate the performance of the proposed method, experiments were conducted on three vehicle tracking datasets, namely, KITTI, UA-DETRAC, and VisDrone2018. The KITTI dataset contains of 21 training sequences and 29 test sequences with more than 19,000 frames [21]. The UA-DETRAC dataset comprises real-world traffic scenes, which includes 60 training and 40 test challenging videos with over 140,000 frames [22]. The VisDrone2018 dataset contains 56 training, 7 validation, and 16 test videos with 5 different categories (car, bus, truck, van, and pedestrian) and 33,366 frames [23].

All those three datasets are challenging in multiple vehicles tracking as they contain large variations in scale, illumination, occlusion, background clutter of scenes, and various type of vehicles. To make a fair comparison with several state-of-the-art (SOTA) multiple object tracking methods, the publicly available detections [23–25] that are recommended by the KITTI, UA-DETRAC, and VisDrone2018 datasets are used in multi-object tracking.

### 4.2. Parameter Settings and Implementation Details

The proposed method is implemented using python language in PyTorch framework, and the network is trained on an Nvidia GTX 2080Ti GPU. The pubic available detections are cropped and resized into 128 *∗* 64 pixels and are then fed into the feature extractor (Resnet-50) to generate the feature maps *f*{*·*}. Then the features *f*{*·*} go through a 1 *∗* 1 convolution layer and are flattened to form patch tokens for two-stage transformer encoder module as described in Section 3.2. The temporal length of tracklets *T* is five in the temporal transformer encoder module, and the feature embedding dimension *C* is 1024. The STE module and TTE module have same architecture design. The MHA block has eight heads and MLP has two layers. Adam optimizer in [26] with an initial learning rate 1e-4 is used in training. The learning rate drops by a factor of 10 at 100 epochs, and the training lasts 180 epochs. The other hyper-parameter setting and training strategy is following ViT [27].

For quantitative evaluation, the metrics defined in [28, 29] are adopted. These metrics are multiple object tracking precision (MOTP)↑, multiple object tracking accuracy (MOTA)↑, fragment (FG)↓, ID-switch (IDs)↓, false positive (FP) ↓, false negative (FN) ↓and the mostly-tracked (MT) ↑, mostly-lost (ML) ↓metrics. For metrics with (↑), the higher values denote better performance. For metrics with (↓), the lower values are better.

### 4.3. Ablation Studies

To better explore the effectiveness of the proposed method, ablation studies are carried out to analyse the effect of each component. Here, the KITTI training set is split into a training set with 10 sequences and a validation set with 11 sequences. The ablation analysis is performed on the validation set.

First, to know how the temporal length of tracklets *T* in the temporal transformer encoder model influences the tracking performance, we set *T*=1, 10, and 15, respectively (the default setting in this paper is *T*=5). It can be seen from the evaluation results in Table 1, when *T*=10 and 15, the MOTA values are 3.9% and 3.7% higher than the values when *T*=1, respectively. *T*=1 indicates that only current tracked object is associated with the detections, and no temporal history trajectory information is introduced in the encoder stage. As shown in Table 1, the tracking performances of other methods when *T*=10 and 15 are worse than those our method with *T*=5. A higher *T* means not only more trajectory information is involved, but also the complexity for data association is increased. Additionally, as defined in data association, a tracked object will be killed if it is not updated more than five consecutive frames. Hence, the strategy of increasing number of *T* does not gain tracking performance; this is consistent with the results in Table 1.

To further analyze the influence of the object queries and track queries for improving the performance of the proposed method, object queries and track queries are separately performed in ablation studies and are defined as P1 and P2 trackers, respectively. From the results shown in Table 2, when only the object query is used as input of spatial transform decoder model, the data association is implemented among the object queries and the detection bounding boxes. Thus, the P1 tracker achieves 84.3% MOTA, which is inferior to that of P2 tracker. This is due to the fact that, in the P1 tracker, no history trajectory information is used to guide the data association in consecutive frames. When the tracked object moves in a small area, the model can correctly associate the detections and the tracked objects. Otherwise, the tracked objects move through a wide area, and this model fails to associate. In the P2 tracker, only the tracker query is used as input of the spatial transform decoder model. Then the data association is performed among the track queries and the detections; the P2 tracker achieves 86.5% MOTA. With the history tracklets information introduced in data association, it is able to associate the objects moved in a wide area. However, the low FN indicates that various objects are missed. The is caused by the fact that the P2 model can only track the objects belonging to the set of tracklets; it ignores the new born ones. With the default setting, the proposed method achieves 88.4% MOTA. By combining the object queries and track queries in our work, all of the above cases can be addressed with the help of two-stage transformed encoder model and spatial transform decoder model.

### 4.4. Comparison with the State-of-the-Art Trackers

#### 4.4.1. Evaluation on KITTI Dataset

Table 3 shows the tracking result of the proposed method compared with the 15 SOTA trackers on KITTI-car testing sequences. The 15 SOTA trackers include six offline trackers and nine online ones. The results demonstrate that the proposed tracking method achieves competitive performance among all online and offline trackers, with the highest MOTA value of 86.9% and MT value of 83.1%. The relatively higher metrics of MOTA and MT and the lower metrics of the ML, IDS, and FG demonstrate that the proposed method can effectively track the vehicles with fewer false negatives proving the good robustness of the proposed model. The proposed method encodes the spatial correlation and temporal history trajectories information at the image level and tracklet level, which effectively extract context information from the tracklets and detections. Furthermore, the image-level and tracklet-level information from the two-stage transformer encoder module is fed back to guide association affinity matrix computation in spatial transformer decoder module. This is useful for using historical tracklets information to handle the occlusion in online tracking.

Figure 4 shows typical vehicle tracking results of the proposed method in handling the occlusion on the KITTI dataset. Each row in Figure 4 shows the tracked vehicles from the same sequence. The tracked vehicles are identified by different color bounding boxes and the identity numbers for the tracked targets are only used for reference. From the 0014 sequence in Figure 4(a), the identity 1 with 90-degree scale changes and the vehicle with identity 1 undergoes occlusion from partial to full. When identity 1 is fully occluded by identity 2 in frame 584, only the latter is tracked. However, when the full occlusion disappears, the proposed method correctly tracks each of them. In 0015 and 0017 sequences, the vehicles with identity number 1 both suffer from occlusion, scale, and illumination changes. When the full occlusion occurs in frames 581 and 119 of sequences 0015 and 0017, the proposed method can only track the vehicles with identity number 2 in both sequences. When the occlusion disappears, the proposed method can successfully associate the occluded vehicle to its previous trajectory in frames 594 and 123 of sequences 0015 and 0017, respectively. These three tracking examples show that the proposed method can effectively tackle the challenges, such as occlusion, scale, and illumination changes, demonstrating its robustness.

#### 4.4.2. Evaluation on UA-DETRAC Dataset

Table 4 presents the quantitative tracking and comparison results of the proposed method with other 9 SOTA trackers on UA-DETRAC dataset. It is seen from Table 4 that the evaluation metrics are heavily influenced by the detectors. When the proposed tracker is tested on CompACT detector, the value of MOTA is 20.14%. For the RCNN detector, the MOTA value is 20.82%. Similar results are obtained for the DCT and IOU trackers as shown in Table 4. These results further validate that the tracking performance is heavily affected by the quality of detections. Additionally, since UA-DETRAC is a challenging dataset in real-world traffic scenes with various traffic crossing, serious occlusion, and different weather conditions, the detections provided by predefined detectors have poor quality, resulting in the MOT metrics, such as MOTA, MOTP, and MT, to be generally inferior to the KITTI datasets for all trackers. Despite this, the overall performance of our tracker is superior to that of other trackers, as shown in Table 4.

Figure 5 shows the typical tracking results of the proposed method on the UA-DETRAC. Similar to Figure 4, each row in Figure 5 shows the tracked vehicles from the same sequence and are identified by different color bounding boxes. Identity numbers are used for reference. From the MVI_40853 sequence, identity 2 is occluded by identity 1, from partial to full. When identity 2 is partially occluded by identity 1 in frame 381, the proposed method can correctly track each one. However, the full occlusion occurs in frame 423, in which only identity 1 is tracked. When the occlusion disappears in frame 463, the proposed method can correctly reidentify identities 1 and 2. Sequence MVI_40763 is a night-time traffic scene. As shown in Figure 5(b), the tracked vehicles are heavily affected by reflected light. Identity 1 is occluded by identity 2 from frames 410 to 442. When the full occlusion happens in frame 449, identity 1 cannot be tracked. A similar phenomenon occurs for identities 2 and 3. When the former is fully occluded by the latter, only identity 3 is tracked. In frame 463, when identity 2 is redetected, the proposed method can successfully associate this vehicle to its previous trajectory. These examples show that the proposed method can handle the occlusion and successfully reidentify the occluded target, validating its robustness.

#### 4.4.3. Evaluation on VisDrone2018 Dataset

To further evaluate the effectiveness of the proposed method, we conduct experiment on VisDrone2018 dataset, which is also a challenging MOT dataset captured from different cities under various weather and lighting conditions. VisDrone2018 dataset mainly focuses on pedestrian, car, van, bus, and truck.  Table 5 presents the comparison results of the proposed method with other 10 SOTA trackers on VisDrone2018 dataset. As shown in Table 5, the proposed tracker has superior tracking performance to other trackers, with 40.5% MOTA. The relatively higher metrics of MOTA and MT and the lower metrics of the ML, IDS, and FG demonstrate the proposed method can effectively track the objects with fewer false negatives, which further validate the effectiveness of the proposed spatial-temporal encoder-decoder affinity network designed for MOT. With the two-stage transformer encoder module, the spatial correlation and temporal history trajectories features at the image level and the tracklet level are fully captured, which is useful for eliminating track errors caused by occlusion. Furthermore, the self-attention and position mechanism in transformer model further help the proposed network to focus on more important features by computing attention weights for object query and tracklet query and to feed the results into the spatial transformer decoder module for association affinity computation, which is beneficial to gain the tracking performance.

### 4.5. Run-Time Performance

The speed of the trackers is evaluated on the UA-DETRAC dataset and VisDrone dataset by frame per second (FPS). The run-time performance of the proposed method and other state-of-the-art trackers are compared in Tables 6 and 7. The run-time for the proposed method is measured on Intel Core i7 16 GHz PC, which is without code optimization and parallel programming. It is seen from Tables 6 and 7 that the run-time performance of the tracker in our method is above the average of all the listed state-of-the-art trackers. Despite this, the speed is insufficient for real-time application. Real-time MOT considering both the validation and speed should be paid more attention to in the future.

### 4.6. Limitation and Future Research

Although the proposed method can be correctly tracking multiple vehicles online, it still needs to be improved until it can be used in real applications. Firstly, the proposed method uses an offline predefined detector to provide the detections; it is not trained for a given traffic video, which may limit the vehicles tracking performance. Hence, how to design a customization object detector and adaptively introduced it into MOT is one of the important directions for our future work. Secondly, the proposed method mainly focuses on how to exploit the powerful representation ability and attention mechanism of deep neural network to model the spatial and temporal relationship of the tracklets and the detections; no extra motion information has been introduced in data association. The motion model learned from data can be used to predict trajectory of the tracked object, which is essential for accomplish track association in situation such as occlusion and tracked objects with similar appearance. Therefore, how to design a unified framework to efficiently construct data association model to make different features (appearance model, motion model) from the tracklets and the detections be compatible with each other is another work that needs to be done in future. Thirdly, although the proposed method is online tracking, the run time is only 8.3 FPS, which is slow for the real-time application. Therefore, real-time MOT should be paid more attention to in our future work. Additionally, in real urban traffic scenarios, the traffic congestion will cause serious occlusion or object disappear issue. Recent development reidentification (Re-ID) model is a good way to solve the occlusion and the target disappeared in surveillance video. Therefore, how to efficiently embed Re-ID model into MOT framework for better solving the occlusion or tracked target disappeared issue is another issue that needs to be solved in the future.

## 5. Conclusion

In this study, we have explored a spatial-temporal encoder-decoder affinity network for multiple vehicle tracking. To fully exploit the spatial and temporal information of the tracked objects in different frames for association affinity computation, a two-stage transformer encoder module is devised to encode candidate detections and the tracked targets for capturing the spatial correlation and temporal history trajectories features at the image level and tracklet level. With the two-stage transformer encoder module, the proposed method can effectively learn the features by leveraging the superiority of the transformer models, where the self-attention and position mechanism focus on more important features by computing attention weights for object query and tracklet query. Moreover, instead of exploiting the spatial and temporal features separately in computing association affinity, a spatial transformer decoder module is designed to compute the association affinity with the feedback results from the two-stage transformer encoder module. This is useful for fully capturing and encoding the spatial and temporal information from the detections and the tracklets of tracked targets. The experimental results compared with state-of-the-art tracker on three benchmark vehicle tracking datasets including KITTI, UA-DETRAC and VisDrone2018 demonstrate that the proposed method has good tracking performances with higher MOTA, MT and lower ML, IDs metrics, validating the effectiveness of the proposed method. We hope that our work will encourage more investigations of exploiting the transformer's powerful attention mechanism for further improving performance of multiple object tracking.

## Figures and Tables

**Figure 1:** Framework of the proposed method.

**Figure 2:** Spatial transformer encoder module for image-level feature extraction.

**Figure 3:** Spatial transformer decoder module for computing association affinity matrix.

**Figure 4:** Tracking examples of the proposed method on KITTI dataset. (a) Sequence 0014. (b) Sequence 0015. (c) Sequence 0017.

**Figure 5:** Tracking examples of the proposed method from UA-DETRAC dataset. (a) Sequence MVI_40853. (b) Sequence MVI_40763.

**Table 1:** Different lengths of tracklets for temporal transformer encoder model on KITTI validation.

Method	FP↓ (%)	FN↓ (%)	MOTA↑ (%)
*T*=1-tracker	8.9	10.1	83.2
*T*=10-tracker	5.3	5.8	87.1
*T*=15-tracker	5.5	6.1	86.9
Ours	5.2	5.9	88.4

**Table 2:** Different input queries for spatial transformer decoder model on KITTI validation set.

Method	FP↓ (%)	FN↓ (%)	MOTA↑ (%)
P1-tracker	7.9	9.4	84.3
P2-tracker	6.4	7.1	86.5
Ours	5.2	5.9	88.4

**Table 3:** KITTI dataset evaluation results.

Dataset	Method	Setting	MT↑ (%)	ML↓ (%)	IDS↓	FG↓	MOTA↑ (%)	MOTP↑ (%)
KITTI Car	MCMOT_CPD [30]	Offline	52.31	11.69	228	536	78.90	82.13
	DSK [31]	Offline	60	8.31	296	868	76.15	83.42
	Complexer-YOLO [32]	Online	58	5.08	1186	2092	75.7	78.46
	NOMT [33]	Offline	41.08	25.23	31	207	66.6	78.17
	LP_SSVM [34]	Offline	35.54	21.26	62	539	61.77	76.93
	CEM [35]	Offline	20	31.54	125	396	51.94	77.11
	RMOT [36]	Online	21.69	31.859	209	727	52.42	75.18
	ODAMOT [37]	Online	27.08	15.54	389	1274	59.23	75.45
	SCEA [38]	Online	26.92	26.62	104	448	57.03	78.84
	CIWT [39]	Online	13.75	34.71	112	901	43.37	71.44
	FAMNet [40]	Online	51.38	8.92	123	713	77.08	78.79
	SASN-MCF [41]	Online	58	7.85	443	975	70.06	82.65
	MASS [42]	Online	74	2.92	353	516	84.64	85.36
	SAMT [43]	Online	62.77	6.00	198	294	83.64	85.89
	CenterTrack [24]	Online	82.15	2.46	254	227	88.83	84.97
	Ours	Online	83.1	2.9	271	254	86.90	85.71

**Table 4:** UA-DETRAC dataset evaluation results.

Dataset	Method	Setting	Detector	MT↑ (%)	ML↓ (%)	IDS↓	FG↓	MOTA↑ (%)	MOTP↑ (%)
UA-DETRAC	GOG [44]	Offline	CompACT	13.90	19.90	3334.6	3172.4	14.20	37.00
	H2T [45]	Offline	CompACT	14.8	19.4	852.2	1117.2	12.40	35.7
	IHTLS [46]	Offline	CompACT	13.8	19.9	953.6	3556.9	11.10	36.8
	DCT [47]	Offline	CompACT	6.7	29.3	141.4	132.4	10.80	37.1
	DCT [47]	Offline	R-CNN	10.1	22.8	758.7	742.9	11.7	38.0
	CEM [34]	Offline	CompACT	3	35.3	267.9	352.3	5.10	35.2
	CMOT [48]	Online	CompACT	16.1	18.6	285.3	1516.8	12.60	36.1
	IOU [49]	Online	CompACT	14.8	19.7	2308.1	3250.4	16.10	37.0
	IOU [49]	Online	R-CNN	13.8	20.7	5029.4	5795.7	16.00	38.3
	V-IOUT [50]	Online	CompACT	17.4	18.8	363.8	1123.5	17.7	36.4
	FAMNET [40]	Online	CompACT	17.1	18.2	617	970.2	19.80	36.7
	Ours	Online	CompACT	17.6	18.1	518.2	1546.8	20.14	34.37
	Ours	Online	R-CNN	18.9	17.6	463.4	1450.6	20.82	35.65

**Table 5:** VisDrone2018 dataset evaluation results.

Dataset	Method	Setting	MT↑	ML↓	IDS↓	FG↓	MOTA↑ (%)	MOTP↑ (%)
VisDrone2018	H2T [45]	Offline	214	494	1269	2035	32.2	73.3
	IHTLS [46]	Offline	245	446	1435	2662	36.5	74.8
	GOG [44]	Offline	244	496	1114	2012	38.4	75.1
	CEM [35]	Offline	105	752	1002	1858	5.1	72.3
	CMOT [48]	Online	282	435	789	2257	31.5	73.3
	SCTrack [51]	Online	211	550	798	2042	35.8	75.6
	TBD [52]	Online	302	419	1834	2307	35.6	74.1
	V-IOUT [50]	Online	297	514	265	1380	40.2	74.9
	Ctrack [53]	Online	369	375	1376	2190	30.8	73.3
	FRMOT [23]	Online	254	463	1043	2534	33.1	73.0
	Ours	Online	319	451	779	2090	40.5	74.1

**Table 6:** Run-time performance (FPS) with different object detector on UA-DETRAC dataset.

Trackers		GOG [44]	H2T [45]	DCT [47]	CEM [35]	IOU [49]	Famnet [23]	CMOT [48]	TBD [52]	IHTLS [46]	Ours
FPS	CompACT	389.51	3.02	2.19	4.62	100.84	0.6	3.79	4.88	19.79	7.5
	RCNN	352.8	2.78	0.71	5.4	—	—	3.59	3.17	11.96	8.3

**Table 7:** Run-time performance (FPS) on VisDrone dataset dataset.

Trackers	H2T [45]	IHTLS [46]	GOG [44]	CEM [35]	CMOT [48]	SCTrack [51]	TBD [52]	V-IOUT [50]	Ctrack [53]	FRMOT [23]	Ours
FPS	1.56	16.3	564.8	7.74	1.39	2.9	0.7	20	15	5	8.3

## Data Availability

The KITTI dataset is available at http://www.cvlibs.net/datasets/kitti/eval_tracking_overview.php. The UA-DETRAC dataset is available at https://detrac-db.rit.albany.edu
